The article "The Balance Reaction Ability of Teenagers Based on the Evaluation Model of Unbalanced Sports Quotient" was retracted in 2023. Reasons: signs of a paper mill; compromised peer review; unreliable results or conclusions.

# The Balance Reaction Ability of Teenagers Based on the Evaluation Model of Unbalanced Sports Quotient

**DOI:** 10.1155/2022/5639893

**Published:** 2022-07-30

**Authors:** Xiwen Yang, Ruihua He

**Affiliations:** ^1^Pingxiang University, Pingxiang, 337055 Jiangxi, China; ^2^Hebei University of Engineering, Handan, 056038 Hebei, China; ^3^Adamson University, Philippines

## Abstract

Dynamic balance is particularly important for the maintenance, transformation, and restabilization of various postures of the human body. Combined with the characteristics of unbalanced sports events, although there is no physical contact in sports events, it has intense antagonism due to the constant change of body movement. Athletes need to have the ability of fast movement and continuous high-intensity multibeat confrontation. They need to adjust their body posture any time according to the situation, constantly move their body from one side to the other side in fast movement, and constantly change between being imbalanced and being stable to keep the center of gravity stable and adjust their body posture. Combining with the characteristics of unbalanced sports, this paper is aimed at the problem that young athletes have poor dynamic balance ability and cannot maintain the stability of their body's center of gravity in the process of fast multidirectional movement and braking. The supporting leg needs ankle dorsiflexion, knee flexion, and hip flexion during SEBT testing. Therefore, the lower limb needs sufficient range of motion, strength, proprioception, and neuromuscular control ability to achieve the optimal test results. A randomized controlled experiment was used to test whether there were significant differences in the test indicators between the experimental group and the control group before and after the experiment by using a paired test. The test indicators between the experimental group and the control group before and after the intervention were tested by independent sample test to explore the influence of core balance training on the dynamic balance ability of teenagers in unbalanced sports. Through analysis, it is proved that strengthening balance exercise can significantly improve the functional movements and physical fitness of adolescents, which is of great significance to the development of basic flexibility and stability of joints and the strengthening of weak chain muscles.

## 1. Introduction

Balance ability refers to the ability of the body to quickly adjust its posture in a specific posture or under the action of external forces and to maintain this posture, reflecting the ability of the human body to coordinate and synthesize stimuli from vestibular organs, muscles, tendons, proprioceptors in joints, and vision. The balance ability is mainly affected by vestibular receptors, muscle strength, vision, and proprioceptors. Intervention training on related factors can improve balance ability. For example, visual intervention training can improve the balance ability of Taijiquan practitioners [1–2].

Literature [3] demonstrated in the study that the explosive force and maximum strength quality of lower limbs have been significantly improved. It can be seen that resistance training of lower limbs has a good effect on improving the strength of swimmers' lower limbs because the strength of lower limbs is related to the improvement of core stability. Literature [4] found that the training method can improve the balance ability of middle school Latin dancers after 8 weeks of static balance ability test, dynamic balance ability test, and core torsion training for 20 students in the experimental group. It also strengthens the cohesion of the core muscles of the players, regulates the psychological stability of middle school students, and improves the body shape. It is a training method with professional pertinence, innovation, and practicability. On the one hand, it broadens the vision of middle school students and helps them enrich their professional knowledge. On the other hand, it improves their interest in learning, which is conducive to adjusting their body and mind and enhancing their psychological stability in the sensitive stage of adolescence. Literature [5] has designed a set of balance training in the study of the influence on the development of students' balance technology, which mainly includes the use of front and back foot position standing posture, left and right foot standing posture, split leg standing, and heel raising exercises. After 12 weeks of auxiliary exercises, it was found that the training could improve students' balance skills, enhance the cohesion of core muscles, improve the range of reflexive confrontation, and adjust the ability of psychological stability. During the exercise, the progress of concentration in the inner thigh and the middle of the body would be increased, which was conducive to improving the core stability of the body. It improves the balance ability of the body and the stability of the trunk and realizes the effective transmission of movements. The main purpose is to relieve muscle fatigue and soreness, avoid the accumulation of lactic acid, roll and massage through foam shafts and other equipment, accelerate the blood circulation of soft tissues, and improve the rate of metabolism to relax the muscles [6].

Balance training in an unstable state is an effective supplement to the traditional balance training in a stable state. Balance training in an unstable state can activate the activities of deep muscle groups and small muscle groups with low excitability and recruit more motor units. It can improve the ability of the central nervous system to control body posture and better meet the needs of modern tennis training [7]. At present, there is little research on the balance ability of male students in tennis classes in China and there is a lack of balance ability training combined with tennis in an unstable state [8]. Therefore, it is becoming a trend to use the training of balance ability under unstable states to design-related balance ability.

In this paper, the body balance training is introduced into the physical quality training of teenagers, which will be conducive to improving the dynamic balance ability of teenagers, enhancing sports quality in training, giving full play to stable technology, and finding suitable teaching methods to enhance the physical quality for the course of body control balance. At the same time, it provides a practical basis for the wide application of core balance training in physical education. Through experimental analysis, there is a significant positive correlation between core balance-related test indicators and dynamic balance ability. The improvement of core balance is conducive to improving the dynamic balance level of sports participants and plays an important role in improving the efficiency of dynamic balance.

The main innovations of this paper are as follows:

1. Exploring the influence of balance training on teenagers' stability ability enriches the theory and method of special balance ability training and also makes a new attempt to the rationality and effectiveness of special balance ability training means
2. The SPSS 19.0 software was used for data analysis. The independent sample *t*-test was used for analysis between groups. The paired sample *t*-test was used for analysis within groups according to the size of the *P* value to analyze whether there is a significant difference or not and draw relevant conclusions

## 2. Object and Method of the Study

### 2.1. Study Object

The experimental team selected 30 members aged 9–11 years. Thirty players were divided into an experimental group and a traditional training group by drawing lots. Fifteen players in the experimental group received functional training three times a week, while 15 players in the traditional training group received traditional training three times a week. To ensure the effectiveness of the experiment, the basic situation of 30 members of the long training class who participated in the experiment was investigated before the beginning of the experiment and it was found that 30 members of the long training class were in good physical condition, without diseases and sports injuries [9]. The basic information of the experimental team members is shown in Table 1.

In Table 1, there was no significant difference in age, height, and weight between the experimental group and the traditional training group before the experiment, *P* > 0.05. It shows that the grouping of the two groups is reasonable and the experimental intervention can be carried out on the two groups of players [10].

### 2.2. Arrangement and Control of the Experiment

#### 2.2.1. Determination of Training Time

The time of a training session is established according to the recommendations in the ACSM Exercise Test and Exercise Prescription Guidelines [11], which recommends that the training time of a session for adolescents should be 60 minutes, of which the initial and final time should be controlled at 5–10 minutes [12]. Therefore, this experiment finally determines that the training time of a class is 60 minutes. The initial part is 10 minutes. The basic training part is 40 minutes, and the end part is 10 minutes. See Tables 2 and 3 for the training course arrangement of the experimental group and the traditional training group.

## 3. Motion Evaluation Model

### 3.1. Initial Stage

Because the experimental team members have not undergone systematic physical fitness training, the initial stage is the initial stage. Firstly, nerve activation, dynamic stretching, and muscle mobilization are the initial activities. The main purpose is to wake up sleeping muscles, prevent sports injuries, and enhance proprioceptors. Then, it is to learn the basic movements of functional training, mainly to develop trunk strength exercises for full support of the body, followed by the gradual development of upper and lower limb strength exercises, which are mainly to improve the coordination ability of the body and develop basic strength [13]. The training program for the initial stage is shown in Table 4.

### 3.2. Advanced Stage

After the basic exercises in the initial stage, a certain intensity is increased based on the basic exercises in the initial stage and the quality of movement completion is emphasized. By strengthening the mobilization level of muscle movement units, more and deeper muscles can be recruited to participate in body movement and improve the strength of small muscle groups [14]. The movement is still the same as in the initial stage. By continuing to practice, the team members can quickly enter the basic part of the exercise state and awaken the deep muscles. In trunk support training, the difficulty and intensity of the exercises are enhanced. Swiss balls, minibelts, balance discs, and other equipment are added to the equipment. The main purpose of adding this equipment is to improve the ability of athletes to maintain balance and stability in an unstable state. The fast telescopic compound training is still used for the trunk and upper and lower limbs. To make body movements more coordinated, this stage requires a higher nervous system [15]. The training scheme for the advanced stage is shown in Table 5.

### 3.3. Consolidation Phase

After two stages of training, the body balance, joint flexibility, and body symmetry of 15 players in the experimental group have been improved and improved to some extent. Therefore, the functional training in the consolidation stage will be more specialized. At this stage, we need to continue to strengthen the practice of trunk support, and at the same time, we need to combine with special skills. Trunk support training from the beginning of four-point support and three-point support to the present two-point support and ball support, through the series and superposition of movement patterns, as well as the coordination of upper and lower limbs and the whole body movement patterns, can better improve the transmission efficiency of the power chain. At this stage, more emphasis is placed on the combination with the special movement to match the sports goals, so the functional training of the special movement mode is also added [16]. The training program for the consolidation phase is shown in Table 6.

### 3.4. Traditional Training Programs

Traditional training only pays attention to single physical fitness training and most exercises with various resistance forces. It is believed that the key to improving the special ability is to improve the strength of muscles, especially the strength of large muscle groups, single muscles, and single joints. In that case, the physical fitness of athletes can be improved [17]. The specific training arrangements are as follows:

#### 3.4.1. Initial Phase

The initial stage is mainly to make the body start systematic physical fitness training. At this stage, the load intensity of training should not be too large, mainly to improve the basic physical fitness of the body [18]. The training scheme for the initial stage of traditional training is shown in Table 7.

#### 3.4.2. Basic Stage

After the initial stage of practice, on the basis of the basic exercises in the initial stage, a certain amount of intensity has been added, mainly to strengthen the exercise of muscle strength and physical coordination. It is required to maintain good movement quality and improve practice efficiency in the training process [19]. The training scheme for the initial stage of traditional training is shown in Table 8.

#### 3.4.3. Consolidation and Improvement Stage

After the first two stages of training, the physical quality of the traditional training group members has been improved to a certain extent. On the basis of consolidating the first two stages of training, the consolidation stage will carry out consolidation muscle strength training to develop muscle endurance and explosive power in an all-round way [20]. The training program for the consolidation phase of traditional training is shown in Table 9.

## 4. Analysis on the Test Results of Balance Reaction Ability

When the human body is in motion or under the action of external forces, the balance response ability can make the human body automatically adjust its posture and control its center of gravity to achieve the optimization of movement control, which is one of the basic sports abilities of the human body. Especially in sports, athletes need to constantly change their positions and movements and the body's center of gravity often changes between imbalance and stability [21]. Combining with the characteristics of unbalanced sports events, this paper holds that balanced reaction ability is an important part of sports ability. In this study, the eight-point star offset balance test with similar multidirectional movement characteristics and high reliability and validity was used to evaluate the balance reaction ability of the experimental team members.

### 4.1. Comparison of Test Results of Balance Reaction Ability of Experimental Team Members

In the eight-point star offset balance test, all the pretest indexes of the experimental team members obey the normal distribution. Before the formal start of the experiment, an independent sample *t*-test was conducted on the standardized values of the pretest indicators of the SEBT test, which effectively evaluated the balanced response ability of the experimental group and the traditional training group. The results are shown in Table 10.

The distance between the traditional training group and the experimental group in the outer front direction of the right leg support is significantly higher than that of the left leg support, and there is a significant difference (*P* < 0.01). The distance between the traditional training group and the experimental group in the inner back direction of the right leg support is significantly higher than that of the left leg support, and there is a significant difference (*P* < 0.05) as shown in Figure 1 [22].

There is an imbalance in the balance reaction ability of the left and right sides of the experimental team members. Studies have shown that when the distance between the left and right sides is more than 4 cm, compensatory movements are more likely to occur in sports. The risk of injury will be 2.5 times higher than that of practitioners with more balanced development on both sides [23].

### 4.2. Comparison of Test Results of the Balance Reaction Ability of Experimental Team Members

After 8 weeks of core balance training, the SEBT test results of the left and right legs of the two groups of experimental players were compared again, as shown in Table 11.

The extension distance of the traditional training group in the front, outer front, and inner direction of the right leg support was significantly higher (*P* < 0.05) than that of the left leg support. After 8 weeks of core balance training, the test results of the SEBT test on the left and right legs, including the comprehensive performance, were similar and the difference (*P* > 0.05) was not significant, as shown in Figure 2.

Core balance training has a positive impact on the coordinated development of the balance reaction ability of the left and right sides of the practitioners. Compared with the traditional training group, it will produce less compensatory movements in sports, which will greatly reduce the risk of sports injury and play a positive role in the prevention of the sports injury [24].

### 4.3. Comparison of Test Results of Balance Reaction Ability in the Traditional Training Group

After 8 weeks of general physical fitness training, the traditional training group used the paired sample *t*-test to compare the SEBT test results before and after training, as shown in Table 12.

Compared with before training, only the extension distance in the lateral direction under left leg support and right leg support has significant difference (*P* < 0.05). Although the test results in other directions and comprehensive performance under left leg support or right leg support have slightly improved, they are not statistically significant (*P* > 0.05). It shows that traditional physical fitness training is not obvious to improve the balance reaction ability of practitioners.

### 4.4. Comparison of the Results of the Balance Reaction Ability Test

After 8 weeks of core balance training, the results of the SEBT test after the experimental group were compared by the paired sample *t*-test, as shown in Table 13.

The experimental group, whether under the support of the left leg or the right leg, has a significantly higher performance in all directions and comprehensive results than the test results (*P* < 0.05) as shown in Figure 3.

The difference between the lower front, outer front, outer back direction, and comprehensive performance of the left leg support and the lower lateral direction and comprehensive performance of the right leg support is the most significant (*P* < 0.01). It can be seen that the core balance training program in this study is conducive to improving the level of balance response of practitioners.

## 5. Conclusion

In this paper, by referring to the SEBT training, based on combining the characteristics of unbalanced sports, progressive balance training is designed. The purpose is to enrich the teaching methods of teenagers' body balance and ultimately to improve the level of teenagers' physical fitness. The results of the SEBT test in all directions and comprehensive performance were significantly higher than those before intervention (*P* < 0.05). Compared with the traditional physical fitness training group, the results of the SEBT test in all directions and comprehensive performance were significantly improved (*P* < 0.05), except the left leg support in the lower front and lateral direction. The right leg support in the lower lateral and medial front direction had no significant difference. Experimental analysis shows that the improvement of teenagers' dynamic balance ability is more significant and it is also conducive to the balanced development of students' dynamic balance ability on both sides. In sports, especially in the intense confrontation of noncontact and high-intensity sports, it helps to strengthen the ability of posture control and maintain the stability of the center of gravity. It also provides a theoretical reference for the research of other related fields.

In this study, an 8-week core balance training program was adopted. Although it can effectively improve the core balance of practitioners, to make the training effect of core balance more significant in the latter study, it is suggested that the training time should be extended appropriately. The training intensity should be increased, the efficiency of the core balance of practitioners should be improved, and the fulcrum should be created for upper and lower limb movement, which is to optimize the generation, transmission, and control of force.

## Figures and Tables

**Figure 1:** Comparison of SEBT test results between the left and right sides of the experimental team.

**Figure 2:** Comparison of SEBT test results between the left and right sides of the team members.

**Figure 3:** Comparison of SEBT test results of experimental groups.

**Table 1:** Basic information of experimental team members.

Indicators	Experimental group	Traditional training group	*T* value	*P* value
Age	11.25 ± 1.52	11.74 ± 1.73	0.000	1.000
Height	152.14 ± 4.74	151.58 ± 4.78	0.155	0.901
Weight	42.93 ± 5.08	43.54 ± 5.15	−0.258	0.741

**Table 2:** Design and arrangement of training courses for the experimental group.

Parts	Time (minutes)	Training contents	Training objectives
Functional initial training component	10	Initial activity, muscle activation	Overcome physiological inertia, and reduce the occurrence of sports injuries
Functional basic training component	40	Depending on the training at each stage	Complete training tasks and achieve training objectives
		Task-based functional movement training	—
End section	10	Functional stretching	Stretch and relax

**Table 3:** Design and arrangement of training courses for the traditional training group.

Parts	Time (minutes)	Training contents	Training purpose
Initial training component	10	Initial activity, jogging	Warm up
Traditional training component	40	According to the different training of each stage; traditional training for the task	Complete training tasks and achieve training objectives
End section	10	General relaxation	Tensile relaxation

**Table 4:** Training program in the initial stage.

Practice forms	Practice action	Required equipment	Amount of exercise	Intermission time
Initial action	Run in small steps	Rope ladder	3 times × 2 groups	5 s
	Quick pad run	Rope ladder	3 times × 2 groups	5 s
	Tuck your knees and raise your heels	Bare hands	5 times × 2 groups	5 s
	Sumo squat	—	5 times × 2 groups	5 s
	Split squat	—	5 times × 2 groups	5 s

Torso strut	Prone T	—	10 times × 3 groups	25 s
	Push-ups	—	10 times × 2 groups	35 s
	Sit-ups	—	15 times × 2 groups	25 s
	Supine hip bridge	—	30 seconds × 3 groups	35 s
	Knee flexion and hip abduction	—	20 times × 3 groups	25 s
	Rotate left and right abdominal muscles at hip	—	30 times × 2 groups	25 s

Quick expansion and contraction compound	Squat jump in place	Bare hands	10 times × 2 groups	25 s
	Jump sideways on both legs	—	10 times × 2 groups	25 s

Recovery and regeneration	Lower limb muscles relax, trunk muscles relax	Foam shaft, massage stick	—	—
	Relaxation, trigger point massage	Static stretching	10	None

**Table 5:** Training plan for the advanced stage.

Practice forms	Names of practice action	Required equipment	Excise amount	Intermittent
Initial action	Cross jump back and forth	—	25 s × 2 groups	5 s
	Moving in and out	Rope ladder	3 times × 2 groups	5 s
	Tuck your knees and go	—	5 times × 2 groups	5 s
	Front lunge stretch	—	5 times × 2 groups	5 s
	Sumo squat	—	5 times × 2 groups	5 s

Torso strut	Single-leg plank	—	25 s × 2 groups	35 s
	Swiss ball curl	Swiss ball	10 times × 3 groups	25 s
	Swiss ball-pinch ball turn hip	Swiss ball	10 times × 3 groups	25 s
	Balance disk squat	Balance disk	30 times × 2 groups	25 s
	The V starts at both ends	Minibelt	20 times × 2 groups	35 s
	Rotate left and right abdominal muscles at hip	—	30 times × 3 groups	25 s

Quick expansion and contraction compound	Explosive push-ups	Bare hands	10 times × 2 groups	25 s
	Leapfrog continuously on both feet	—	10 times × 2 groups	25 s

Recovery and regeneration	Muscles relax loosen, trigger massage	Foam shaft, massage stick, yoga mat	10	None

**Table 6:** Training programs for the consolidation phase.

Practice forms	Action practice	Required equipment	Amount of exercise	Intermission time
Initial action	Fast footwork in place	—	25 s × 2 groups	5 s
	Moving in and out	Rope ladder	3 times × 2 groups	5 s
	Minibelt lateral forward	—	10 times × 2 groups	5 s
	Creeper	—	5 times × 2 groups	5 s
	Sumo squat	—	5 times × 2 groups	5 s

Torso strut	Plank (with one hand and one foot)	—	10 times × 2 groups	25 s
	BOST ball upper elbow brace	BOST ball	30 seconds × 2 groups	35 s
	Swiss ball up	Swiss ball	10 times × 2 groups	25 s
	Hanging push-up	Elastic band	10 times × 2 groups	35 s
	Fold your legs, pull in your knees, and turn your hips to ski	Swiss ball	10 times × 2 groups	25 s
	Single-leg support abduction	Swiss ball	10 times × 2 groups	25 s

**Table 7:** Initial training program of the traditional training group.

Practice forms	Action practice	Amount of exercise	Intermission time
Initial activity	Jogging	800 m	2 minutes
	Head and neck exercises	4 × 8 beats	None
	Shoulder joint movement	4 × 8 beats	None
	Body rotation movement	4 × 8 beats	None
	Knee joint movement	4 × 8 beats	None
	Wrist and ankle exercises	4 × 8 beats	15 s

Basic parts	Hand and foot support	10 seconds × 2 groups	25 s
	Sit-ups	10 times × 2 groups	25 s
	Supine static leg lift	20 seconds × 2 groups	25 s
	Jump on one or both feet	30 seconds × 3groups	35 s
	Half squat	10 times × 2 groups	25 s
	Stand up and squat	10 times × 3 groups	25 s
	Run back and forth	20 meters × 2 groups	35 s

Relaxation activities	Jumping jacks	30 times × 2 groups	25 s
	Wrist stretch, abdominal stretch, leg stretch	10	None

**Table 8:** Training program for the traditional training group in the initial stage.

Practice forms	Movement training	Amount of exercise	Intermission time
Initial activity	Jogging	800 m	2 minutes
	Head and neck exercises	4 × 8 beats	None
	Shoulder joint movement	4 × 8 beats	None
	Body rotation movement	4 × 8 beats	None
	Knee joint movement	4 × 8 beats	None
	Wrist and ankle exercises	4 × 8 beats	15 s

Basic parts	Plank support	30 seconds × 2 groups	25 s
	Lie on your back and get up at both ends	15 times × 2 groups	25 s
	Lie prone and back up	10 times × 3 groups	25 s
	Skipping exercise	1 min × 2 groups	1 minute
	Kneeling jump	10 times × 2 groups	25 s
	Lunge forward	10 times × 3 groups	25 s
	Squat	15 times × 2 groups	25 s

Relaxation activities	Run with high legs	20 meters × 2 groups	35 s
	Wrist stretch, abdominal stretch, leg part stretch	10	None

**Table 9:** Training program for the consolidation phase of the traditional training group.

Practice forms	Movement training	Amount of exercise	Intermission time
Initial activity	Jogging	800 m	2 minutes
	Head and neck exercises	4 × 8 beats	None
	Shoulder joint movement	4 × 8 beats	None
	Body rotation movement	4 × 8 beats	None
	Knee joint movement	4 × 8 beats	None
	Wrist and ankle exercises	4 × 8 beats	15 s

Basic parts	Push-ups	15 times × 2 groups	35 s
	Plank support	30 seconds × 2 groups	35 s
	Quickly start at both ends	30 times × 2 groups	1 min
	Bobby jump	10 times × 2 groups	1 min
	Quick high leg lift in place	30 seconds × 3 groups	35 s
	Leapfrog	10 times × 2 groups	25 s
	Weight-bearing lunge	10 times heart group	25 s

Relaxation activities	Squat and curled knee jump	20 times × 2 groups	25 s
	Wrist stretch, abdominal stretch, leg stretch	10	None

**Table 10:** Comparison of SEBT test results of two groups of experimental team members (*N* = 15) (cm).

Supporting leg	Indicators	Traditional training group (*N* = 8)	Experimental group (*N* = 7)	*T* value	*P* value
Left leg support	Front	80.5 ± 7.2	83.4 ± 8.1	0.34	0.77
	Outer front	78.5 ± 8.0	75.1 ± 8.2	0.08	0.96
	Outer	68.2 ± 9.6	64.3 ± 10.1	0.62	0.65
	Outer back	82.4 ± 11.2	82.9 ± 10.6	−0.09	0.94
	Back	87.4 ± 11.1	90.4 ± 10.4	−0.41	0.61
	Inner back	85.3 ± 11.4	91.1 ± 10.9	−0.89	0.39
	Inner	81.2 ± 10.1	95.3 ± 10.3	−0.91	0.44
	Inner front	90.3 ± 9.4	91.5 ± 9.8	−0.21	0.82
	Integrated	84.1 ± 9.3	86.1 ± 10.7	−0.31	0.71

Right leg support	Front	84.7 ± 8.7	85.7 ± 6.9	0.44	0.78
	Outer front	82.3 ± 11.2	71.6 ± 9.7	0.86	0.39
	Outer	67.5 ± 12.5	67.3 ± 10.4	0.11	0.98
	Outer back	81.6 ± 12.7	82.1 ± 11.6	0.12	0.91
	Back	87.2 ± 13.5	91.9 ± 10.7	−0.25	0.88
	Inner back	89.3 ± 12.8	92.6 ± 11.8	−0.35	0.77
	Inner	86.3 ± 11.6	91.3 ± 10.9	−0.31	0.76
	Inner front	88.1 ± 9.7	91.5 ± 9.8	−0.09	0.93
	Integrated	82.7 ± 11.1	85.1 ± 12.7	0.06	0.87

**Table 11:** Comparison of SEBT test results of two groups of experimental team members (*N* = 15) (cm).

Supporting leg	Indicators	Traditional training group (*N* = 8)	Experimental group (*N* = 7)	*T* value	*P* value
Left leg support	Front	81.6 ± 6.6	92.2 ± 6.5	−2.05	0.06
	Outer front	78.3 ± 6.8	85.3 ± 5.9	−3.09	0.01
	Outer	77.6 ± 8.7	86.9 ± 8.7	−0.42	0.42
	Outer back	88.8 ± 5.5	93.0 ± 6.1	−3.36	0.02
	Back	88.4 ± 9.2	93.3 ± 7.3	−2.42	0.03
	Inner back	92.1 ± 9.3	97.6 ± 8.6	−2.41	0.03
	Inner	88.6 ± 7.9	98.0 ± 6.3	−2.63	0.03
	Inner front	93.5 ± 3.1	92.7 ± 3.7	−2.83	0.02
	Integrated	87.2 ± 6.4	96.8 ± 6.8	−2.98	0.02

Right leg support	Front	88.3 ± 4.5	96.1 ± 1.2	−2.75	0.03
	Outer front	77.2 ± 3.4	88.0 ± 3.1	−3.88	0.01
	Outer	73.6 ± 7.7	87.4 ± 10.6	−1.24	0.22
	Outer back	86.8 ± 5.3	92.3 ± 5.9	−3.65	0.01
	Back	92.1 ± 4.6	91.5 ± 6.7	−2.82	0.01
	Inner back	93.5 ± 4.0	93.4 ± 5.2	−3.64	0.02
	Inner	91.5 ± 2.5	90.3 ± 6.1	−2.73	0.02
	Inner front	92.6 ± 6.8	95.7 ± 3.0	−2.18	0.02
	Integrated	86.9 ± 4.7	91.1 ± 5.8	−2.84	0.05

**Table 12:** Comparison of SEBT test results in the traditional training group (*N* = 8) (cm).

Supporting leg	Indicators	Traditional training group	Experimental group	*T* value	*P* value
Left leg support	Front	85.4 ± 8.8	84.2 ± 6.7	1.53	0.11
	Outer front	76.8 ± 8.7	72.3 ± 6.5	−0.64	0.52
	Outer	69.9 ± 12.1	78.6 ± 8.6	−4.75	0.05
	Outer back	84.2 ± 13.8	89.8 ± 5.2	−1.17	0.27
	Back	88.7 ± 12.7	84.9 ± 9.6	−0.55	0.56
	Inner back	87.6 ± 12.7	92.1 ± 9.6	−1.50	0.12
	Inner	87.9 ± 12.8	84.4 ± 7.9	−1.02	0.31
	Inner front	90.3 ± 8.7	98.9 ± 3.1	−1.46	0.27
	Integrated	83.7 ± 11.5	89.3 ± 6.8	−1.57	0.11

Right leg support	Front	85.8 ± 8.7	83.3 ± 4.3	−0.51	0.62
	Outer front	81.0 ± 14.4	72.1 ± 3.6	1.02	0.35
	Outer	66.5 ± 12.5	76.3 ± 7.4	−3.14	0.06
	Outer back	82.4 ± 11.6	85.2 ± 5.6	−1.48	0.11
	Back	88.6 ± 10.3	90.8 ± 4.4	−0.76	0.42
	Inner back	88.8 ± 10.8	91.8 ± 4.1	−1.01	0.34
	Inner	87.7 ± 10.5	95.6 ± 2.2	−1.44	0.15
	Inner front	89.8 ± 9.8	93.9 ± 6.6	−0.77	0.40
	Integrated	83.1 ± 11.2	85.4 ± 4.8	−1.29	0.24

**Table 13:** Comparison of SEBT test results of posttest groups (*N* = 7) (cm).

Supporting leg	Indicators	Traditional training group	Experimental group	*T* value	*P* value
Left leg support	Front	84.7 ± 7.5	91.2 ± 6.4	−8.26	0.01
	Outer front	76.5 ± 7.7	82.3 ± 5.5	−11.34	0.01
	Outer	66.2 ± 10.4	83.9 ± 8.6	−6.03	0.01
	Outer back	84.0 ± 11.6	97.0 ± 6.1	−4.35	0.02
	Back	92.4 ± 12.4	92.3 ± 7.7	−3.24	0.03
	Inner behind	95.3 ± 13.3	97.6 ± 8.8	−2.64	0.05
	Inner	92.4 ± 10.9	98.0 ± 6.2	−2.78	0.04
	Inner front	90.2 ± 7.1	94.7 ± 3.3	−2.76	0.05
	Integrated	85.3 ± 10.2	92.8 ± 6.4	−4.73	0.01

Right leg support	Front	84.0 ± 8.9	93.1 ± 1.7	−3.46	0.00
	Outer front	77.1 ± 10.1	87.0 ± 3.6	−3.78	0.01
	Outer	65.4 ± 11.2	80.4 ± 10.7	−8.51	0.01
	Outer back	81.8 ± 10.8	91.3 ± 5.3	−3.83	0.02
	Back	90.6 ± 11.4	92.5 ± 6.5	−3.77	0.03
	Inner back	91.6 ± 10.7	96.4 ± 5.4	−2.75	0.01
	Inner	90.4 ± 12.6	94.3 ± 6.6	−2.63	0.02
	Inner front	90.7 ± 10.4	96.7 ± 3.8	−2.72	0.03
	Integrated	83.9 ± 10.3	97.1 ± 5.9	−4.04	0.01

## Data Availability

The data used to support the findings of this study are available from the corresponding author upon request.
